The article "Laparoscopic versus Conventional Surgery for Acute Cholangitis of Severe Type: A Systematic Review of Randomized Controlled Trials" was published in 2022. Journal: Comput Math Methods Med.

# Laparoscopic versus Conventional Surgery for Acute Cholangitis of Severe Type: A Systematic Review of Randomized Controlled Trials

**DOI:** 10.1155/2022/6828476

**Published:** 2022-06-16

**Authors:** Fang Zhang, Jianjiang Huang, Jie Yang, Yuyu Wang, Bin Qiu

**Affiliations:** Critical Care Medicine, Shengzhou People's Hospital (The First Affiliated Hospital of Zhejiang University Shengzhou Branch), Zhejiang Province 312400, China

## Abstract

**Objective:**

Currently, the choice between laparoscopic surgery and conventional laparotomy in the surgical treatment of acute cholangitis of severe type (ACST) is debatable. This study compared the clinical efficacy of these two surgical methods through a meta-analysis based on relevant clinical randomized controlled trials (RCT) on ACST.

**Methods:**

We systematically searched several databases (PubMed, Web of Science, Embase, China National Knowledge Infrastructure, and WangFang) for RCT on the surgical treatment of ACST between 2010 and 2022. Relevant data were extracted, and a meta-analysis was performed using the statistical software Stata 16.0.

**Results:**

From initial 1089 studies retrieved, 15 studies (*n* = 1247 patients) were eligible. The total number of patients was 1247, of whom 635 were classified in the treatment group (laparoscopic surgery) and 612 patients in the control group (conventional laparotomy). This meta-analysis showed that compared with conventional laparotomy, laparoscopic surgery was associated with higher effective rate (OR = 3.808, 95% CI [2.383, 6.085], *P* < 0.001), lower incidence rate of complications (OR = 0.192, 95% CI [0.139, 0.265], *P* < 0.001), shorter operation duration (SMD = −3.274, 95% CI [-4.503, -2.045], *P* < 0.001), and shorter postoperative hospital stay (SMD = −2.432, 95% CI [-2.988, -1.877], *P* < 0.001). Further, the indicators of symptomatic relief (anus exhaust time, jaundice relief time, gastrointestinal function recovery time, and abdominal pain relief time) and inflammatory levels (white blood cell count, alanine aminotransferase, total bilirubin level, and high-sensitivity C-reactive protein level) in the treatment group were better than those in the control group.

**Conclusion:**

Laparoscopic surgery was associated with significant improvement in treatment efficiency, reduced risk of complications, and better treatment outcomes in patients with ACST.

## 1. Introduction

Acute cholangitis (AC) is defined as acute suppurative inflammation caused by ascending bacterial infections of the biliary tract. Specifically, biliary stones can induce sudden biliary obstruction, leading to cholestasis, elevated pressure, and infection in the biliary tract and ultimately reflux of bacteria into the blood [1]. AC is characterized by an acute onset, rapid progression, and high mortality rate [2]. According to the Tokyo Guidelines (TG13/18) for severity grading [3], AC combined with the presence of cardiovascular, neurological, respiratory, hematologic, renal, or hepatic dysfunction could be classified as AC of severe type (ACST). Moderate AC is diagnosed when two of the following symptoms are present: abnormal white blood cell count (WBC), high fever, age ≥ 75 years old, hyperbilirubinemia, and hypoalbuminemia. ACST, also known as acute obstructive suppurative cholangitis (AOSC), is the most severe among different grades. It can progress rapidly and can have a high mortality rate unless timely treatment is provided [4]. Currently, the surgical maneuver for biliary surgery of ASCT remains challenging.

The 2018 Tokyo Guidelines (TG18) [5], interpreted by Hu et al., recommend that moderate to severe AC should be treated with urgent biliary drainage (BD), in addition to antibiotics, to relieve biliary hypertension caused by biliary obstruction and to avoid the entry of bacteria and toxins into the bloodstream, which could otherwise result in inflammatory cascades. Additionally, bile duct stones causing cholangitis must be removed after the improvement of the patient's condition. Clinically, safe biliary decompression can safely follow within 24 hours of antibiotic use, adequate resuscitation, and stabilization of organ function [6]. Early surgical treatment has been shown to reduce fatalities [7]. BD was previously performed surgically but has also been associated with a high mortality rate due to large trauma and high requirement for postoperative nursing. In recent years, with the advancement of endoscopic technology, endoscopic BD, including percutaneous transhepatic cholangial drainage (PTCD), endoscopic sphincterotomy (EST), and endoscopic nasobiliary drainage (ENBD), are currently the recommended types of surgery for treating ACST. ENBD and PTCD can be performed laparoscopically at the same time. The combination of duodenoscopy, laparoscopy, and choledochoscopy has been shown to reduce trauma and surgical procedures, thereby facilitating postoperative recovery and achieving better clinical results in elderly ACST patients [8, 9]. However, some studies have revealed that EST combined with ENBD could also result in bleeding, acute pancreatitis, and even perforation, and the operation and proficiency of surgeons are highly demanded [10]. Thus, the choice of surgical methods for treating ACST remains debatable.

In this study, we systematically retrieved relevant randomized controlled trials (RCTs) comparing conventional surgery versus laparoscopic treatment for ACST and performed a meta-analysis to evaluate their therapeutic effects and associated posttreatment levels of inflammatory-related markers. We hope that these findings could provide evidence and guidance for the surgical management of ACST.

## 2. Materials and Methods

### 2.1. Search Strategy

PubMed, Web of Science, Embase, China National Knowledge Infrastructure, and WangFang databases were searched to identify randomized controlled trials (RCTs) comparing conventional surgery versus laparoscopic treatment for ACST from 2010 to 2022. The keywords used included “acute cholangitis of severe type” AND “laparoscopic surgery” OR “surgery”.

### 2.2. Inclusion and Exclusion Criteria of Studies

The study inclusion criteria were as follows: (1) study design: clinical RCTs published in medical journals at home and abroad; (2) study subjects: patients diagnosed with ACST or AC according to the guidelines for diagnosis and treatment of acute biliary tract infections (2021) [11]; (3) intervention measures: treatment group consisted of laparoscopic surgery, while the control group consisted of traditional laparotomy; and (4) outcome measures: at least with any one of the following parameters: effective rate, incidence rate of complications, duration of surgery, postoperative hospital stay, time to symptomatic recovery (i.e., anal exhaust, jaundice relief, gastrointestinal function recovery, abdominal pain relief), and inflammatory factor levels (WBC, alanine aminotransferase (ALT), total bilirubin (Tbil), and high-sensitivity C-reactive protein (hs-CRP)).

The study exclusion criteria were as follows: (1) study design or intervention measures inconsistent with the topic of this meta-analysis; (2) original studies failed to provide relevant data required for this meta-analysis; (3) duplicate literature; and (4) literature with ambiguous diagnostic criteria or outcome measures.

### 2.3. Literature Screening and Data Extraction

The literature titles retrieved were imported into the Endnote 7.0 software to eliminate repeated ones. Then, two investigators independently screened the literature to extract the data and evaluate the quality of the retrieved literature in strict accordance with the inclusion and exclusion criteria. In case of any dispute, a third investigator was consulted for consensus. The data extracted mainly included the following: title, name of the first author, study design, intervention measures, patient baseline data, eradication rate of Hp, and incidence of adverse events. The risk of bias of the included articles was evaluated using the assessment tool recommended in Cochrane Handbook 5.1.0.

### 2.4. Statistical Analysis

The Stata 16.0 statistical software was used for meta-analysis. Odds ratio (OR) and corresponding 95% confidence interval (CI) were used to express enumeration data, while continuous variables were expressed as standardized mean difference (SMD) and 95% confidence interval (CI). Heterogeneity among the results of each study was assessed using the chi-square test and *I*^2^ statics. The fixed effects model was applied for comparisons without statistical heterogeneity among the studies (*P* > 0.05 and *I*^2^ ≤ 50%); otherwise, the random effects model was used for analysis. *P* < 0.05 was considered statistically significant.

## 3. Results

### 3.1. Basic Information of the Included Studies

Initially, 1089 articles were retrieved. After excluding 147 duplicated articles and 422 unqualified, 505 articles failing to meet the inclusion criteria were also excluded after reading their full text. Finally, 15 RCTs were included in this meta-analysis [12–26], comprising 1247 patients (treatment group: laparoscopic surgery, *n* = 635; control group: traditional laparotomy, *n* = 612). The literature screening process is shown in Figure 1. The characteristics of the included studies are displayed in Table 1. The included articles were evaluated for quality using the assessment tool provided in the Cochrane Handbook (Figures 2(a) and 2(b)).

### 3.2. Clinical Effects of Laparoscopic Surgery in the Treatment of ACST

#### 3.2.1. Meta-Analysis Results of Response Rate and Incidence of Complication after Treatment

Twelve studies compared the treatment response rate after surgery in patients with ACST, and 15 studies reported the incidence of complications after treatment. There was no significant heterogeneity among the studies (treatment response rate: *I*^2^ = 0.0%, *P* = 0.958; incidence rate of complications: *I*^2^ = 0.0%, *P* = 0.869), and the fixed effects model was taken for analysis. The study results showed that the effective rate of laparoscopic surgery for ACST was significantly higher than that of conventional laparotomy (OR = 3.808, 95% CI [2.383, 6.085], *P* < 0.001; Figure 3(a)), and the incidence rate of complications was significantly lower than that of conventional laparotomy (OR = 0.192, 95% CI [0.139, 0.265], *P* < 0.001; Figure 3(b)).

Further, sensitivity analysis was performed for the effective and incidence rates of complications (Figures 4(a) and 4(b)). The results were consistent with the *P* value, *I*^2^ value, and OR of the original meta-analysis results, showing no significant difference and indicating good stability of the meta-analysis results. Subsequently, publication bias analysis was performed, and an asymmetric distribution was observed in the funnel plots (Figures 4(c) and 4(d)). Such distribution indicated that the included studies had a certain level of publication bias, which could be related to the small sample size of some studies or the low quality of the included literature.

#### 3.2.2. Meta-Analysis Results of Duration of Surgery and Postoperative Hospital Stay

Nine articles compared the duration of surgery, and 13 studies compared the postoperative hospital stay between the two groups. The random effects model was used to combine the effect sizes (operation duration: *I*^2^ = 97.4%, *P* < 0.001; postoperative hospital stay: *I*^2^ = 92.1%, *P* < 0.001). The results showed that compared with laparotomy, laparoscopic surgery was associated with shorter operation duration (SMD = −3.274, 95% CI [-4.503, -2.045], *P* < 0.001; Figure 5(a)) and postoperative hospital stay (SMD = −2.432, 95% CI [-2.988, -1.877], *P* < 0.001; Figure 5(b)).

Sensitivity analysis was performed to identify the source of heterogeneity, and the random effects model was used for analysis. The results were consistent with the *P* value, *I*^2^ value, and OR of the original meta-analysis results, showing no significant difference and indicating good stability of the meta-analysis results (Figures 5(c) and 5(d)).

#### 3.2.3. Meta-Analysis Results of Symptom Relief Indicators

Five articles reported on anal exhaust time, gastrointestinal function recovery time, and abdominal pain relief time, and four articles reported on jaundice relief time. The effect sizes of three of the four indicators were combined using the random effects model (anal exhaust time: *I*^2^ = 99.2%, *P* < 0.01; jaundice relief time: *I*^2^ = 73.7%, *P* = 0.010; and abdominal pain relief time: *I*^2^ = 86.1%, *P* < 0.001), and one was analyzed using the fixed effects model (gastrointestinal function recovery time: *I*^2^ = 45.4%, *P* = 0.120). Our meta-analysis revealed that compared with the control group, patients who underwent laparoscopic surgery required shorter time to achieve anal exhaust (SMD = −5.188, 95% CI [-9.757, -0.619], *P* = 0.026, Figure 6(a)), jaundice relief (SMD = −0.807, 95% CI [-1.216, -0.399], *P* < 0.001, Figure 6(b)), gastrointestinal function recovery (SMD = −1.221, 95% CI [-1.482, -0.960], *P* = 0.04, Figure 6(c)), and abdominal pain relief (SMD = −2.431, 95% CI [-3.079, -1.783], *P* < 0.001, Figure 6(d)) after treatment.

Further, sensitivity analysis was performed. The results were consistent with the *P* value, *I*^2^ value, and OR of the original meta-analysis results, showing no significant difference and indicating good stability of the meta-analysis results (Figures 6(e)–6(h)).

#### 3.2.4. Meta-Analysis Results of Inflammatory Factor Indicators

Four RCTs reported on WBC and ALT levels, and Tbil and hs-CRP levels were mentioned in five studies. Compared with the control group, laparoscopic surgery was associated with lower postoperative levels of WBC (SMD = −0.943, 95% CI [-1.366, -0.521], *P* < 0.001; Figure 7(a)), ALT (SMD = −2.469, 95% CI [-3.620, -1.317], *P* < 0.001; Figure 7(b)), Tbil (SMD = −2.709, 95% CI [-2.969, -2.448], *P* < 0.001; Figure 7(c)), and hs-CRP (SMD = −2.514, 95% CI [-3.395, -1.633], *P* < 0.001; Figure 7(d)). Further, sensitivity analysis showed low sensitivity of WBC (Figure 7(e)), ALT (Figure 7(f)), Tbil (Figure 7(g)), and hs-CRP (Figure 7(h)) levels, indicating that the results of this meta-analysis were robust and credible.

## 4. Discussion

Biliary obstruction caused by intrahepatic and extrahepatic bile duct stones, biliary stricture, or biliary ascariasis can result in hypertension and infection of the biliary tract infection, ultimately leading to bile reflux and bacteria into the blood and ACST [27]. Therefore, relieving obstruction via surgical biliary decompression and drainage is necessary to avoid further systemic organ injury and improve treatment outcomes [28]. Laparoscopic surgery was introduced in the treatment of biliary tract diseases because of its small incisions and good prognosis. Additionally, the surgical procedures are fewer, and the duration of surgery is shorter in laparoscopic surgery compared with laparotomy. A multicenter retrospective study by Sugiura et al. [29] observed that the probability of dysfunction in malignant hilar biliary obstruction using ENBD was 26.5%. Theoretically, laparoscopic surgery for ACST has shown good efficacy, but there is a lack of effective evidence, so exploring the actual effects of laparoscopic surgery for ACST could guide physicians to better plan surgical treatment.

This meta-analysis included 15 studies with a total of 1247 patients. According to the results, for patients with ASCT, laparoscopic surgery was associated with a higher effective rate, lower incidence of complications, and better performance of symptom relief and inflammation after treatment. These findings are consistent with the results of Hu, wherein endoscopic surgery was found to be significantly better than laparotomy in terms of abdominal pain disappearance time, off-bed activity time, incidence of complications, and hospital stay [30]. Traditional surgical treatment is invasive, needs more time to complete and longer recovery time, and could affect the recovery of patients, especially elderly and frail patients who have a poor tolerance to surgery due to diminished physiological function, and could thus lead to a higher risk of complications. With developments in endoscopic technology and minimally invasive surgeries, lesser invasive surgical strategies have the advantages of less trauma, quick recovery, and improved treatment outcomes [31, 32].

Clinically, WBC, CRP, and Tbil levels and imaging findings are usually used as diagnostic and prognostic evaluations for AC [33]. The results of this study showed that WBC, Tbil, hs-CRP, and ALT levels in patients with ACST treated with laparoscopic surgery were markedly improved than those in those treated with traditional laparotomy. Our results concur with those of Li et al. [34], in which laparoscopic surgery was shown to be more conducive to postoperative inflammatory recovery in acute and severe cases than laparotomy, suggesting that the former could indeed reduce the risk of toxins entering the blood circulation and the spread of inflammation.

## 5. Conclusion

Compared with traditional laparotomy, laparoscopic surgery demonstrated good clinical efficacy in patients with ACST. Laparoscopy was associated with lesser trauma and faster recovery. Specifically, laparoscopic surgery had the advantages of shorter operation duration, lower incidence of complications, less postoperative inflammatory response, and shorter hospital stay. Thus, laparoscopy could be considered a safe and effective treatment method for patients with ACST, providing the theoretical basis to guide surgeons in making clinical decisions on the surgical management of these patients.

## Figures and Tables

**Figure 1:** Flowchart of literature screening.

**Figure 2:** (a) Distribution of risk of bias in the retrieved literature. (b) Literature risk assessment results.

**Figure 3:** Forest plots comparing the clinical efficacy in the two groups of patients with ACST: (a) treatment response rate; (b) incidence rate of complications after treatment.

**Figure 4:** Sensitivity analysis and funnel plot of clinical efficacy in the two groups of patients with ACST: (a, b) sensitivity analysis of treatment response rate (a) and incidence of complications after treatment (b); (c, d) funnel plots of treatment response rate (c) and incidence of complications after treatment (d).

**Figure 5:** Forest plots and sensitivity analysis of operation duration and postoperative hospital stay: (a, b) sensitivity analysis of operation duration (a) and postoperative hospital stay (b); (c, d) funnel plots of operation duration (c) and postoperative hospital stay (d).

**Figure 6:** Forest plots and sensitivity analysis of symptom relief indicators in the two groups of patients with ACST: (a–d) forest plots of postoperative anal exhaust time (a), jaundice relief time (b), gastrointestinal function recovery time (c), and abdominal pain relief time (d); (e–h) sensitivity analysis of postoperative anal exhaust time (e), jaundice relief time (f), gastrointestinal function recovery time (g), and abdominal pain relief time (h).

**Figure 7:** Forest plots and sensitivity analysis of postoperative inflammatory factors in the two groups of patients with ACST. (a–d) Forest plots of WBC (a), ALT (b), Tbil (c), and hs-CRP (d); (e–h) sensitivity analysis of WBC (e), ALT (f), Tbil (g), and hs-CRP (h). WBC: white blood count; ALT: alanine aminotransferase; Tbil: total bilirubin; hs-CRP: high-sensitivity C-reactive protein.

**Table 1:** Basic characteristics of the included literature.

Study	Year	Sample time	Group	Cases	Age (years)	M/cases	Study design	Outcome measures
Li Xiaodong [6]	2012	2007/01-2010/12	Treat	42	71.96 ± 11.86	26	RCT	(1)(2)(3)(4)(12)
			Cont	35	73.02 ± 9.53	20		
Li Junyao [7]	2017	2013/06-2016/06	Treat	44	70.1 ± 10.9	25	RCT	(1)(2)(4)(6)(7)(8)
			Cont	44	72.1 ± 8.9	20		
Luo Yang [8]	2019	2016/01-2017/12	Treat	72	72.5 ± 6.6	39	RCT	(1)(2)(3)(4)(5)(6)(7)(8)(11)
			Cont	72	71.8 ± 6.4	40		
Cheng Xianchen [10]	2018	2014/03-2018/01	Treat	28	70 ± 3.1	15	RCT	(1)(2)(3)(4)(5)
			Cont	28	76.5 ± 4.5	12		
Wang Yuepin [11]	2017	2014/03-2016/03	Treat	42	26-75	22	RCT	(1)(2)(3)(4)(5)(9)(10)
			Cont	42	26-75	23		
Wu Bichuang [12]	2011	2005/06-2010/05	Treat	18	40.5 ± 8.5	7	RCT	(2)(3)(4)
			Cont	19	40.5 ± 8.5	8		
Li Zhiqiang [13]	2020	2015/01-2019/12	Treat	50	56.28 ± 7.85	27	RCT	(1)(2)(4)(7)
			Cont	50	56.42 ± 8.05	26		
Yu Weijun [14]	2013	2009/01-2011/12	Treat	42	65.98 ± 10.83	23	RCT	(1)(2)(3)(4)(5)(9)(12)
			Cont	35	65.98 ± 10.83	24		
Hu Shong [15]	2017	2014/07-2015/02	Treat	46	78.6 ± 6.3	18	RCT	(1)(2)(4)(6)(7)(8)(11)
			Cont	46	78.5 ± 6.4	19		
Feng Rifang [16]	2018	2014/05-2017/05	Treat	54	68.1 ± 7.7	37	RCT	(1)(2)(3)(4)(5)
			Cont	54	68.7 ± 8.1	38		
Liu Yi [17]	2014	2009/11-2012/12	Treat	38	72.0 ± 1.8	23	RCT	(1)(2)(3)
			Cont	38	73.2 ± 2.5	22		
Zhang Yi [18]	2016	2011/01-2015/01	Treat	47	54.53 ± 9.43	19	RCT	(2)(4)(7)(8)(9)(10)(11)(12)
			Cont	35	54.28 ± 0.43	15		
Shen Hongbo [19]	2012	2004/10-2009/10	Treat	45	60-88	29	RCT	(1)(2)(4)(12)
			Cont	56	60-88	32		
Zhou Fan [20]	2015	2009/01-2013/01	Treat	37	73.2 ± 6.6	22	RCT	(2)(6)(8)(9)(10)(11)
			Cont	36	73.2 ± 6.6	21		
He Shi Qing [21]	2013	2010/2-2011/12	Treat	30	67.4 ± 4.8	19	RCT	(1)(2)(3)(4)(10)(11)(12)
			Cont	22	68.3 ± 5.0	14		

Abbreviations: Treat: treatment; Con: control; M: male; RCT: randomized controlled trial. (1) Effective rate; (2) incidence of complications after treatment; (3) operation duration; (4) hospital stay after treatment; (5) anal exhaust time after treatment; (6) jaundice relief time after treatment; (7) recovery time of gastrointestinal function after treatment; (8) duration of abdominal pain relief after treatment; (9) white blood cell count after treatment; (10) alanine aminotransferase level after treatment; (11) total bilirubin level after treatment; and (12) high-sensitive C-reactive protein level after treatment.

## Data Availability

The data used to support the findings of this study are available from the corresponding author upon request.

## Abbreviations

AC: Acute cholangitis
ASCT: Acute cholangitis of severe type
WBC: White blood cell count
BD: Biliary drainage
PTCD: Percutaneous transhepatic cholangial drainage
EST: Endoscopic sphincterotomy
ENBD: Endoscopic nasobiliary drainage
RCT: Randomized controlled trials
ALT: Alanine aminotransferase
Tbil: Total bilirubin
hs-CRP: High-sensitivity C-reactive protein
OR: Odds ratio
CI: Confidence interval
SMD: Standardized mean difference.
